# Artificial Intelligence Algorithm-Based Computed Tomography Images in the Evaluation of the Curative Effect of Enteral Nutrition after Neonatal High Intestinal Obstruction Operation

This article has been retracted.

**DOI:** 10.1155/2021/7096286

**Published:** 2021-11-16

**Authors:** Yanqing Dong, Zhaolong Wang, Zhiguang Zhang, Bobo Niu, Pan Chen, Pengju Zhang, Huizhong Niu

**Affiliations:** Pediatric Surgery, Department of General Surgery, Hebei Children's Hospital, Shijiazhuang 050000, Hebei, China

## Abstract

In this study, CT image technology based on level set intelligent segmentation algorithm was used to evaluate the postoperative enteral nutrition of neonatal high intestinal obstruction and analyze the clinical treatment effect of high intestinal obstruction, so as to provide a reasonable research basis for the clinical application of neonatal high intestinal obstruction. 60 children with high intestinal obstruction treated in the hospital were selected as the research objects. Based on the postoperative enteral nutrition treatment, they were divided into control group (noncatheterization group)-parenteral nutrition support. In the observation group, gastric tube was placed through nose for nutritional support. Then, CT images based on level set segmentation algorithm were used to compare the intestinal recovery of the two groups, and the biochemical indexes and hospitalization were compared. The level set algorithm can accurately segment the lesions in CT images. The segmentation time of the level set algorithm was shorter than that of the traditional algorithm (24.34 ± 2.01 s vs. 75.21 ± 5.91 s), and the segmentation accuracy was higher than that of the traditional algorithm (84.71 ± 3.91% vs. 70.04 ± 3.71%, *P* < 0.05). The weight of children in the observation group (100 ± 7 g) was higher than that in the control group (54 ± 5 g), and the ICU monitoring time (12.01 ± 2.65 days) and the hospital stay (17.82 ± 3.11 days) were shorter than those in the control group (13.42 ± 2.95 days, 19.13 ± 3.22 days, all *P* < 0.05). The level set segmentation algorithm can accurately segment the CT image, so that the disease location and its contour can be displayed more clearly. Moreover, the nasal placement of jejunal nutrition tube can effectively improve the intestinal function of children, maintain the steady-state environment of intestinal bacterial growth, and significantly improve the clinical treatment effect, which is worthy of clinical application and promotion.

## 1. Introduction

Neonatal high intestinal obstruction is mostly caused by organic diseases, such as pyloric diaphragm, pyloric atresia, duodenal stenosis and atresia, annular pancreas, congenital malrotation of the intestine, and other factors [1]. The typical manifestation is vomiting soon after birth. The obstruction is located above the duodenal papilla and the vomit contains no bile. However, if the obstruction is located below the duodenal papilla, the vomit contains no yellow-green bile, the upper abdomen is full, the lower abdomen is flat or the whole abdomen is flat, and the stool is little or no, which requires more surgical treatment [2]. As the birth rate of newborns continues to grow, the incidence rate of high gastrointestinal obstruction is also rising [3]. According to the incidence of neonatal high gastrointestinal obstruction, there are more than 1,500 new cases of congenital high gastrointestinal obstruction in Hebei province every year, and 90% of the children patients need surgical treatment [4]. However, in many provinces, there is no consensus on the treatment of enteral nutrition through jejunal tube for neonatal children with high intestinal obstruction surgery, and the postoperative recovery effect of children patients is uneven due to the lack of standard treatment. Therefore, it is of great clinical, social, and economic significance to summarize the treatment norms of early enteral nutrition for infants with neonatal high intestinal obstruction after postoperative jejunal catheterization [5].

Most of the children patients with timely treatment can improve their disease symptoms, but there are also children patients with deteriorating conditions. Therefore, it is necessary to evaluate the curative effect in time after treatment, so as to make further reasonable and effective countermeasures based on the treatment results [6]. At present, the diagnosis and evaluation of this disease in clinical practice are mainly through plain abdominal X-ray film, but the diagnostic accuracy is not ideal after clinical application [1]. With the continuous development of medical technology, computed tomography (CT) technology has become more and more mature and has been favored by a wide range of medical workers. Many studies have confirmed that abdominal CT examination has a high application value in intestinal obstruction diseases, and the operation is more convenient [7]. In addition, the image data of abdominal CT examination are clearer with higher resolution. Under the premise of good cooperation of the children patients, it can more clearly show the site and severity of the obstruction lesions in the children patients. The enhanced scanning of CT examination method can help clinicians to observe the conditions of the tissues around the lesion from multiple angles and directions, so as to analyze whether the lesions have metastatic signs, thus contributing to accurate evaluation. However, during the scanning process, the child cannot stay still all the time, so there will be motion artifacts in CT imaging. In order to make the result clearer and accurate and facilitate clinical evaluation, the level set algorithm based on the artificial intelligence algorithm was adopted in this study. The target contour of this algorithm is embedded in the distance symbol function of zero level set, so it is necessary to keep the level set function in a good state and make its change curve flatten, so that the evolution process of level set becomes stable and the process of numerical realization is more accurate [8]. Furthermore, level set algorithm helps to accurately define and characterize the spatial range of the region or edge of the target object in the image and improve the recognition. Therefore, it is widely used in the segmentation and processing of CT images of lung, liver, brain, and other diseases [9]. However, the research on CT image technology of level set algorithm in the evaluation of enteral nutrition is relatively lacking.

Therefore, a retrospective study was conducted, 60 children with high intestinal obstruction in the hospital were selected as the research objects, and CT based on level set segmentation algorithm was used to evaluate the therapeutic effect of early enteral nutrition with jejunal intubation and ordinary parenteral nutrition without intubation on children after neonatal high intestinal obstruction, The results provide a scientific and standardized clinical basis for the application of early enteral nutrition in neonatal high intestinal obstruction. By evaluating the quality of clinical trials, we found the shortcomings of current clinical research, and this provided improvement suggestions for further research in the future.

## 2. Materials and Methods

### 2.1. General Data of the Research Objects

60 children patients with high intestinal obstruction admitted to hospital from January 2017 to December 2019 were selected as the research objects. Then, all of them were rolled into the control group and the observation group based on their disease types. Among them, there were 17 male children and 13 female children in the control group; the gestational age range was 38 weeks; the disease distribution was as follows: 14 cases of circular pancreas and 16 cases of duodenal atresia and stenosis. In the observation group, there were 12 male children and 18 female children; the gestational age was 37 weeks; disease distribution was as follows: 19 cases of circular pancreas and 11 cases of duodenal atresia and stenosis. The family members of the patients in this study understood this study and signed the informed consent form. The hospital's medical ethics committee reviewed and approved this study. Diagnostic criteria referred to the relevant diagnostic criteria of high intestinal obstruction in *Ultrasound Diagnosis of Intestinal Obstruction*. The criteria for inclusion were defined to include patients who met the above diagnostic criteria, had the age of admission that was within one month of birth, suffered from congenital intestinal obstructive disease, could receive surgical treatment, and were aware of and signed informed consent by the family members of the children. The criteria for exclusion were defined as follows: those who were combined with other basic diseases that affected feeding; those whose parents did not cooperate with the researcher; those who did not undergo surgical treatment; those who were accompanied with congenital heart disease, etc.

### 2.2. Treatment Methods

The control group (noncatheterized group) received parenteral nutrition support after the surgery, and feeding should be carried out after the children patients' gastrointestinal function was restored. Intravenous nutrition is still given to the child patient to ensure daily physiological requirements until the total feeding energy failed to meet the normal physiological requirements. Besides, intravenous nutrition was discontinued at 105 kcal/kg of calories. The observation group was treated with intraperitoneal jejunal nutrition tube. Moreover, the changes of blood routine, blood biochemical, body weight, and other indicators of the two groups were observed, as well as the differences in the length of hospital stay and hospitalization costs.

### 2.3. CT Image Scanning

Before the examination, the children patients were prepared according to the doctor's advice, and they were injected with pantogluamine (1.5%) through a gastric tube. During the examination, they were placed in the supine position and scanned by a spiral CT scanner with a conventional horizontal axis sweep. Next, the tube current was set to 150 mAs, tube voltage was set to 70 kV, layer thickness was set to 2.4–5.0 mm, layer spacing was set to 2.5–5.0 mm, pitch was set to 1 mm, and matrix was set to 512 × 512. When the ray was transformed into visible light, the photoelectric sensor could be converted into electrical signals, and then the information could be converted into digital signals through the digital-to-analog converter. Finally, the simple computer in CT could be used for operation and reconstruction.

### 2.4. CT Image Processing Based on Artificial Intelligence Algorithm

CT images are processed by intelligent segmentation algorithm, namely, the level set algorithm. The level set algorithm is employed to solve the evolution problems that follow the thermodynamic theory. The flow diagram of the algorithm is shown in Figure 1.

In the level set algorithm, the plane closed curve *Y* can be expressed as an equivalent curve with the same function value of the three-dimensional continuous function surface *I (x, y, z)*, and generally *I* = 0, also called the zero level set, and *I (x, y, z)* is also called the level set function. Then, the position of the zero level set is calculated, and the required contour of the target object can be obtained.

The level set function can be deformed gradually during the evolution process and cannot maintain the distance regularization. Therefore, this research introduced the distance regularized level set evolution (DRLSE) algorithm that would avoid reinitialization. The specific algorithm is as follows. The energy equation for distance regularization is displayed in

(1) $$\begin{array}{c} Q\left(I\right)=iD_{l}\left(I\right)+E_{\text{ext}}\left(I\right), \end{array}$$

where *D*_*l*_(*I*) represents the rule top of the level set, *i* is a constant greater than 0, and *E*_ext_(*I*) means the external energy. Therefore, *D*_*l*_(*I*) can also be defined as follows:

(2) $$\begin{array}{c} D_{l}\left(I\right)\Delta \oint l\left(\left|\Lambda \oint 1\right|\right)sx, \end{array}$$

where *l* stands for the potential energy function, which can not only smooth the evolution of the level set, but also maintain the symbolic distance attribute near the zero level set.

(3) $$\begin{array}{c} l=l_{1}\left(t\right)\Delta \frac{1}{2}{\left(t-1\right)}^{2}. \end{array}$$

When *t* = 1, *l* has a unique minimum point according to

(4) $$\begin{array}{c} l=l_{1}\left(t\right). \end{array}$$

The level set rule top can be expressed in

(5) $$\begin{array}{c} l\left(i\right)=\frac{1}{2}\int {}_{\Omega }{\left(\left|\Delta \oint 1\right|-1\right)}^{2}sx. \end{array}$$

In order to avoid the level set evolution obtained by the minimization of energy from producing undesirable side effects on the level set function *I*, a new potential energy function is introduced.

(6) $$\begin{array}{c} l=l_{2}\left(t\right)=\left\{\begin{array}{c} \frac{1}{2}{\left(t-1\right)}^{2},\;t>1,\\ \frac{1}{{\left(2\Pi \right)}^{2}}\left(1-\cos\left(2\Pi t\right)\right)\left(t\right)1. \end{array}\right. \end{array}$$

Equation (6) maintains the contour of the level set evolution, and the potential energy function has a minimum value at *t* = 1 and *t* = 0.

### 2.5. Statistical Methods

SPSS 21.0 statistical software was used for data analysis. The measurement data were represented by $\bar{x}\pm s$, and *t*-test was performed; count data were expressed as [example (%)], which was for chi-square test; measurement data that met normal distribution were analyzed by variance analysis. For measurement data that did not meet the normal distribution, the rank sum test was employed to analyze the differences between groups; the count data were adopted to analyze the differences between groups by the chi-square test. The Kaplan–Meier method was used to analyze and compare the incidence of adverse events during the follow-up period of the two groups of patients, and the Log-rank test was applied to analyze the differences between the groups. In addition, *P* < 0.05 indicated that the difference was statistically substantial.

## 3. Results

### 3.1. Comparison on Baseline Data between the Two Groups of Children Patients

After comparison, it was found that there was no marked difference in gender and gestational age between the two groups of children patients (*P* > 0.05), as shown in Table 1.

### 3.2. CT Image Examination Results under the Level Set Algorithm

Through image observation and analysis, it was found that the intestinal CT image under the level set algorithm reduced the curve evolution process of the initial level set and avoided the processing of the whole image. Therefore, this algorithm could accurately segment the lesions in the CT image, as shown in Figure 2.

### 3.3. Comparison on Level Set Algorithm and Traditional Algorithm

Figure 3(a) shows the comparison of the segmentation time between the level set algorithm and the traditional algorithm. The segmentation time of the level set algorithm is (24.34 ± 2.01) *s* and that of the traditional algorithm is (75.21 ± 5.91) (*s*). The segmentation time of the level set algorithm is significantly shorter than that of the traditional algorithm.  Figure 3(b) shows the comparison of segmentation accuracy between level set algorithm and traditional algorithm. Among them, the segmentation accuracy of level set algorithm is (84.71 ± 3.91) % and that of traditional algorithm is (70.04 ± 3.71) %. The segmentation accuracy of level set algorithm is significantly higher than that of traditional algorithm (*P* < 0.05).

### 3.4. CT Imaging Examination Results of Children Patients

Figure 4 shows the CT images of two children before and after treatment. A and B are the CT findings of the same child before and after treatment. After treatment, the intestinal torsion of the child is improved, the mesenteric effusion disappears, the air-fluid level phenomenon is significantly reduced, and the symptoms of the child are significantly improved.

### 3.5. The Situation of Children Patients from the Two Groups after Treatment

Figure 5 shows the comparison of the weight, ICU monitoring time, and hospitalization time of the two groups after treatment. The weight of the children in the observation group was (100 ± 7) g and that in the control group was (54 ± 5) g. The monitoring time of children in ICU in the observation group was (12.01 ± 2.65) days and that in the control group was (13.42 ± 2.95) days. The hospitalization time of children in the observation group was (17.82 ± 3.11) days and that in the control group was (19.13 ± 3.22) days. The weight of children in the observation group was significantly higher than that in the control group. The hospital stay in ICU in the observation group was shorter, and the postoperative hospital stay was also shorter than that in the control group (*P* < 0.05).

### 3.6. Results of Routine Blood Tests in Children Patients from the Two Groups

Figure 6(a) shows the changes of total blood protein in the two groups before treatment and 7 days after treatment. The total blood protein in the control group before treatment was (57.12 ± 9.34) g/L and 7 days after treatment was (54.10 ± 6.54) g/(L). The total blood protein of the observation group before treatment was (58.63 ± 6.17) g/L and 7 days after treatment was (52.00 ± 5.23) g/(L).  Figure 6(b) shows the changes of plasma albumin in the two groups before treatment and 7 days after treatment. The plasma albumin in the control group before treatment was (34.37 ± 6.43) g/L and 7 days after treatment was (32.87 ± 4.33) g/(L). The plasma albumin of the observation group before treatment was (36.37 ± 4.55) g/L and 7 days after treatment was (32.64 ± 4.12) g/(L).  Figure 6(c) shows the changes of hemoglobin in the two groups before treatment and 7 days after treatment. The hemoglobin in the control group was (159.41 ± 18.20) g/L before treatment and (121.13 ± 23.45) g/L after 7 days of treatment. The hemoglobin of children in the observation group was (167.87 ± 13.21) g/L before treatment and (115.93 ± 24.56) g/L after 7 days of treatment. Through comparative analysis, the blood protein level of all children patients was improved after treatment. The recovery level of children in the observation group was better than that in the control group, but the protein level of the two groups after 7 days of treatment was not statistically significant (*P* > 0.05).

## 4. Discussion

A newborn is a baby born within 28 days from umbilical cord ligation. Neonatal intestinal obstruction refers to the obstruction of the normal delivery of the contents of the intestinal cavity of the newborn to cause partial or complete failure to pass, resulting in systemic physiological dysfunction [10]. The incidence rate is higher than 1%, which is the main cause of neonatal acute abdomen and one of the important causes of perinatal infant death [11]. The main causes of the disease in children patients are gastrointestinal malformation and dynamic ileus [12]. Embryonic development hypoplasia digestive tract abnormalities in newborns can cause mechanical intestinal obstruction, such as congenital intestinal atresia, congenital intestinal stricture, duodenal atresia, congenital megacolon, congenital intestinal rotation, and intestinal adhesion. In addition, newborns may also cause intestinal peristalsis dysfunction due to abnormal intestinal nerve function and produce dynamic intestinal obstruction [13–15]. Obstruction can occur in any part of the intestine and can be caused by intestinal luminal lesions (fecal block blockage in the intestine) and intestinal wall lesions (intestinal wall inflammation, edema leading to stenosis, intestinal wall tumor, intestinal intusculation or factors outside the intestine, etc.) [16]. After the illness, the child patient will have extremely uncomfortable physical reactions. The main manifestations are abdominal pain, bloating, vomiting, and nondefecation. The symptoms at the onset vary according to the cause of the intestinal paralysis. Newborns may have dyspnea due to abdominal distention, and most of them do not vomit at the early stage. Vomiting occurs after abdominal distention worsens, containing stool-like material, and the frequency of defecation decreases until they cannot exhaust the air [17]. Clinical diagnosis depends on laboratory examinations and imaging examinations. Laboratory examinations include white blood cell count, hemoglobin, hematocrit, carbon dioxide binding capacity, serum potassium, sodium, chloride, urine routine, and stool routine. There are generally no abnormal findings in the early stages of obstruction [18].

Surgical treatment can help children quickly improve adverse symptoms and reduce intestinal pressure [19]. In this study, CT images based on level set segmentation algorithm were used to compare the intestinal changes of children before and after treatment. The results showed that, after treatment, the intestinal torsion of children was improved, the mesenteric effusion disappeared, and the symptoms were significantly improved. This is consistent with the above conclusion. Other studies showed that nutritional support plays an important role in treatment. According to relevant animal experiments, mice with total intravenous nutrition will have intestinal mucosal atrophy, flattened intestinal villi, and blocked lactase development after fasting for only three days, suggesting that enteral nutrition is very important for the integrity of gastrointestinal structure and function [20]. In this study, it was concluded that, after nutritional support treatment, the weight and blood protein level of children in the observation group and the control group were improved, which is consistent with the above conclusions. However, in terms of nutritional support methods in the observation group and the control group, the weight change (100 ± 7) g vs. (54 ± 5) g, ICU monitoring time (12.01 ± 2.65) days vs. (13.42 ± 2.95) days, and hospital stay (17.82 ± 3.11) days vs. (19.13 ± 3.22) days in the observation group were better than those in the control group. Some research data show that early enteral nutrition for newborns with high intestinal obstruction through indwelling nasojejunal nutrition tube is effective, but the selection of milk products and the way of milk volume increase in the process of enteral nutrition are still in the exploratory stage, and the number of domestic relevant studies on the evaluation of their nutritional status is limited [21]. Studies suggested that there is a possibility of concurrent infection with indwelling nasojejunal nutrition [22], which may be different from this study and needs further research.

In order to improve the clarity of images and the integrity of lesions, the level set algorithm in the artificial intelligence algorithm was adopted in this study. In the traditional level set method, the level set function will gradually deviate from the symbolic distance function in the process of evolution, which will cause the instability of the method and result in no error in the image segmentation. It is highly likely that the curve will not converge to the target contour [23]. The usual solution is to use the “reinitialization” method to correct, but the “reinitialization” method will cause new and other problems. These questions may affect the accuracy of the final results; according to the research of experts, the energy function of the level set algorithm model includes the distance normalization term and the external energy that makes the zero level set close to the target contour. However, the distance normalization term is mainly defined and explained by the potential function, and the evolution process of the level set generated by this term can make up for the deficiency of the evolution of the traditional level set. This allows a pull on the level set function to keep it in the ideal shape. The results of this study indicated that the intestinal CT image under the level set algorithm reduced the curve evolution process of the initial level set and avoided the processing of the whole image. The algorithm could accurately segment the lesions in the CT image. The segmentation time of level set algorithm is shorter than that of traditional algorithm, and the segmentation accuracy is higher than that of traditional algorithm (*P* < 0.05), so as to realize the accurate segmentation of CT image. Hoogi (2017) [24] pointed out in the research that the level set algorithm shows significantly better segmentation effect. Compared with the most advanced fixed size local window, the dice similarity coefficient is increased by 0.25 ± 0.13 (Wilcoxon, *P* < 0.001). In addition, the level set algorithm is applied to the segmentation of lung CT. The results show that the CT image based on the algorithm has high accuracy in lung cancer detection, and the sensitivity of the detection algorithm is 91.3%, 96.3%, 80.9%, and 82.3%, respectively [25].

## 5. Conclusion

In conclusion, by using the CT image technology based on the level set intelligent segmentation algorithm to evaluate the postoperative enteral nutrition of newborns with high intestinal obstruction, it is concluded that the level set algorithm can improve the definition of the image, improve the definition of the contour and boundary, and realize the automatic and accurate segmentation of CT images of children with high intestinal obstruction. In addition, it is concluded that nasal insertion of jejunal nutrition tube can effectively improve children's intestinal and digestive functions, reduce intestinal effusion, and maintain a stable environment for intestinal bacterial growth, which is worthy of further clinical promotion. The disadvantage of this study is that it belongs to the central research, and the sample size is small, which has a certain impact on the research results. Therefore, it is necessary to expand the sample size for further research. However, this study clearly reflects the clinical application advantages of nasal jejunal nutrition tube insertion, suggesting that this method has a good application prospect in clinic.

## Figures and Tables

**Figure 1:** Schematic diagram of the level set algorithm flow.

**Figure 2:** CT image examination results under the level set algorithm. (a) Original image. (b) DR-LS algorithm.

**Figure 3:** Comparison on level set algorithm and traditional algorithm. (a) Segmentation time. (b) Segmentation accuracy. ∗ indicates that the comparison is statistically significant (*P* < 0.05).

**Figure 4:** CT imaging examination results of one child patient (the red arrow indicates the original lesion).

**Figure 5:** Comparison on the situation of all the children' patients after treatment. (a) One-week postoperative weight gains. (b) ICU monitoring time. (c) Postoperative hospital stay. ∗ indicates that the comparison is statistically significant (*P* < 0.05).

**Figure 6:** The results of routine blood tests in children patients. (a) Total protein. (b) Albumin. (c) Hemoglobin.

**Table 1:** Comparison on baseline data of children patients from the two groups.

	The number of cases	Gender (male/female)	Gestational age (weeks old)	Age of admission (d)	Age of surgery (d)	The number of cases with annular pancreas	The number of cases with duodenal atresia and stenosis
Control group	30	17/13	38	0	3	14	16
Observation group	30	12/18	37	0	2.5	19	11
*x* ^2^ or *z* value		0.158	1.055	−1.51	0.728	1.684	
*P* value		0.612	0.319	0.1	0.394	0.194	

## Data Availability

The data used to support the findings of this study are available from the corresponding author upon request.
